# Clinical and histopathological characterization of root resorption in replanted teeth: Two case reports

**DOI:** 10.1097/MD.0000000000018869

**Published:** 2020-01-17

**Authors:** Huimin Liu, Xiaoxing Peng, Hongchen Sun, Xiangwei Li

**Affiliations:** a School of Stomatology, Jilin University; b Radiology Department of Hospital Attached to Changchun University of Chinese Medicine, Changchun, PR China.

**Keywords:** periodontal tissue, pulp tissue, replanted permanent teeth, root resorption, trauma

## Abstract

**Rationale:**

The frequency of tooth avulsion is on the rise due to increasing rates of maxillofacial trauma. Avulsed teeth present with varying degrees of root resorption, and are generally asymptomatic; therefore, they often go undiagnosed. The etiopathogenesis of root resorption in replanted teeth following avulsion remains unclear.

**Patient concerns:**

In case 1, the left upper lateral incisor became loose after 10 years of replantation. In case 2, the patient underwent tooth replantation after external root canal treatment due to tooth dislocation caused by trauma 8 years ago.

**Diagnosis:**

According to the medical history, clinical manifestations and imaging studies of the 2 patients, root resorption after replantation was diagnosed.

**Interventions:**

The teeth extraction was given to one patient. Besides the histological examination of extracted teeth was performed.

**Outcomes:**

Teeth that underwent pulp treatment presented with external resorption. On the other hand, the tooth that had received no pulp treatment showed both external and internal resorption; residual vital pulp tissue was detected within the pulp cavity.

**Lessons:**

The dental pulp tissues may be involved in the initiation or development of internal resorption. Trauma to the periodontal ligament might play a major role in external resorption, whereas internal tooth resorption may be caused as a result of injury to the residual pulp tissue. Thus, the effective management of these tissues during the treatment of replanted teeth is essential.

## 1 Introduction

The incidence of tooth avulsion has demonstrated a growing trend following the increases in the rate of maxillofacial trauma.^[1]^ Avulsed teeth with varying degrees of root resorption are generally asymptomatic, and in most cases are found during routine radiographic examinations. Root resorption poses serious deleterious effects on oral function and health, such as weak chewing efficiency,^[2]^ esthetic problems,^[3]^ teeth loss, malocclusion, deficiency of alveolar bone volume, and imperfect facial development.^[4]^

The treatment of an avulsed tooth depends upon the extent and timing of dislocation within the socket. A tooth with a fully developed root can be replaced in its socket immediately following the removal of any contaminants or debris. In some instances, in order to prevent the drying of the tooth, it can be placed in the sublingual or buccal cavity of the patient, or in a cup of milk, saline or water, until further treatment or replantation.^[5]^ Studies show that that root resorption can be avoided in 90% of cases if the avulsed tooth is replanted within 0.5 hours of avulsion, followed by root canal therapy within 3 to 4 weeks of replantation.^[6,7]^

It is important to perform root canal therapy for an avulsed tooth in a timely manner. Trauma to the tooth can result in local pulp necrosis, alveolar damage, traumatic occlusion, and dental resorption. Thus, replantation of an avulsed tooth and subsequent root canal therapy with occlusal adjustments are extremely important. Local pulp necrosis often leads to, or promotes, varying degrees of tooth resorption. In this report, we describe two cases of root resorption in replanted teeth following avulsion due to trauma. The main difference between the two cases was that one patient underwent root canal treatment for the replanted tooth.

Depending on the site, tooth resportion can be classified as internal (wall of root canal) or external (root surface).^[7]^ Internal resorption is further divided into two types: those involving root canal shift, and those presenting with local resorption. Based on various clinical and histological features external resorption is divided into the following four categories: root surface resorption, local resorption on root surface, alternative resorption, and root adhesions.^[8]^ The present report compares the clinical features and resorption patterns between 2 cases of root resorption in replanted teeth following tooth avulsion. We also present the histological observations of an extracted tooth with serious root resorption. The study was approved by the Research Ethics Review Committee of the School and Hospital of Stomatology, Jilin University (Changchun, China). Patients have provided informed consent for publication of the case, and the study was conducted in accordance with the approved guidelines set by the bioethics law of China.

## 2 Case report

### 2.1 Case 1

A 17-year-old male presented with a mobile upper left lateral incisor. History revealed trauma resulting in the avulsion of the upper left central and lateral incisors 10 years ago, which was managed by replantation 2 hours post avulsion. It was noted that root canal treatment had not been performed following replantation. Oral examination revealed significant discoloration of the left maxillary central and lateral incisors when compared with the adjacent teeth. The lateral incisor was mobile (III degree), whereas the central incisor did not show any mobility. The patient did not complain of pain and both teeth were not responsive to hot or cold stimuli. No redness or swelling of the adjacent gingival tissues was observed.

Intra-oral periapical radiographs revealed the presence of several lacunae in the roots of the upper left central and lateral incisors (Fig. 1). Nearly 1/3rd of the root and distal root canal wall of the lateral incisor was resorbed; root fracture was also noticed (Fig. 1). A radiolucency, suggestive of apical periodontitis, was observed in the periapical region. As seen in Figure 1, the distal root surface of the upper central incisor displayed a large lacuna that was connected to the root canal and apical foramen. In addition, a periapical radiolucency was observed in the upper central incisor region (Fig. 1). Clinically, the patients were diagnosed with dental root fracture of the left maxillary lateral incisor and resorption of the left maxillary central incisor. The teeth were cleaned with an oral disinfection reagent and extracted under local anesthesia, which was then followed by thorough curettage of the fossae.

**Figure 1:** Periapical radiograph of replanted upper left maxillary central and lateral incisors. Several lacunae (bold arrows) are seen in the roots of both the central and lateral incisors. Central incisor shows periapical involvement (double arrow), whereas no radiolucency was observed around the periapical region of the later incisor.

### 2.2 Case 2

A 24-year-old male suffering from caries of the central incisors presented with a history of trauma eight years ago, which had resulted in the avulsion of the 2 central incisors for over 2 hours. The avulsed teeth had undergone ex vivo root canal therapy and were subsequently, replanted. No discoloration or mobility of the 2 central incisors was noted on clinical examination. The patient did not complain of pain and both the teeth were not responsive to hot and cold stimuli. The surrounding gingival tissue was also normal.

Further examinations revealed resorption of the distal root canal wall, which had nearly reached the obturation material in the upper right incisor. In the upper left incisor, root resorption was observed on the mesial and distal sides of the tooth in the cervical and middle thirds, leading to the separation of the apical third from the middle third of the root canal. No radiolucency was noted in the periapical region, whereas the surface of the distal root presented with a large lacuna located very close to the obturation material (Fig. 2). The tooth was filled and a subsequent appointment for routine examination was scheduled.

**Figure 2:** Roots of the upper central incisors showing external resorption. The right incisor was resorbed along with the root surface. In the left center incisor, resorbed areas were observed on the distal and mesial profiles of the tooth in the cervical and middle thirds. No radiolucency seen in the periapical regions.

The extracted tooth (lateral incisor) from Case 1 was immediately immersed in 10% neutral-buffered formalin for 48 hours. Demineralization was performed in an aqueous solution containing EDTA, for 4 weeks. The specimen was routine embedded in paraffin. Longitudinal serial sections were made in the mesio-distal plane until the specimen was exhausted. Particular care was taken to obtain and locate sections passing through the foramen. The sections were then stained with hematoxylin-eosin and examined under the light microscope.

The presence of some residual vital pulp tissue was noted in the pulp cavity (Fig. 3A). Several lacunae extending in to the primary dentin were observed in the dentinal walls of the crowns, along with the presence of multinucleated cells (Fig. 3B). Interestingly, in addition to the presence of some odontoblast-containing lacunae, areas of newly formed dentin covering obsolete resorption lacunae were also noted, indicating the simultaneous occurrence of both tooth resorption and regeneration (Fig. 3C). In addition to the few lacunae observed in the portion of the root facing the medullary cavity, a small number of odontoclasts and an abundance of fibroblasts as well as collagen fibers were noted adjacent to the pulp (Fig. 3D). The part of the root facing the periodontal ligament had several lacunae covered by reparative dentin and cementum (Fig. 3E). Granulation tissue present around the apical portion of the roots consisted mainly of fibroblasts, collagen fibers and a large number of lymphocytes. In addition to local hemorrhage and necrosis, local osteoid dentin formation was also noted in the vicinity (Fig. 3F).

**Figure 3:** Micrographs of Hematoxylin and eosin (H&E) stained sections from upper lateral incisor and granulation tissue (Case 1). A: Apical region of the lateral incisor with local pulp necrosis (N), vacuolar changes (V) and vital pulp (P) in the pulp horn (arrow; magnification, 40×). B: Walls of the crowns facing the canal side of the dentin have large numbers of lacunae (L), which extend into primary dentin, where multinucleated cells (double arrow) are observed (100×). C: Some lacunae are seen to be containing odontoblasts (O) with the formation of new dentin (ND), part of which is seen to be covering the obsolete resorption lacunae (100×). D: Observed by light microscopy, there are a few pulp cells, more fibroblasts (F) and collagen fibers in lacunae (100×). E: The part of the root facing the periodontal ligament (PL) consists of several lacunae covered by reparative dentin and cementum (C) (100×). F: Granulation tissue between the ends contained more fibroblasts, collagen fibers (CF) and a large number of lymphocytic (Ly) infiltrates. In addition, local hemorrhage, necrosis, and surrounding local osteoid dentin (OD) formation is noted (100×).

## 3 Discussion

Avulsion is a serious injury of pulp and periodontal tissues. After avulsion and replantation, teeth are at risk of infection and root resorption, which may affect treatment outcome and survival rate. The overall outcome from the meta-analysis showed that the incidence of RR in avulsion was high. The incidence of root resorption after avulsion and replantation in ascending order was internal root resorption < surface root resorption < inflammatory root resorption < replacement root resorption.^[9]^

Clinically, an avulsed tooth with an intact fully developed root should be replaced immediately after thorough removal of all debris within the socket. Resorption can be avoided in nearly 90% of cases if the tooth is replanted within 0.5 hours, followed by root canal therapy within 3 to 4 weeks.^[6,7]^ In cases where the tooth has been dislocated for more than 2 hours, in vitro root canal therapy should be the first stage of treatment, followed by replantation within the socket. Root canal treatment should be performed in all replanted teeth.^[10]^

In the present study, in vitro root canal therapy was not provided to the patient in Case 1, either before or after replantation despite the fact that the teeth had been avulsed for more than 2 hours. Interestingly, both internal and external root resorption ensued along with tissue destruction and root fracture. This implies that residual dental pulp and periodontal ligament cells, which may have experienced hypoxia and severe dryness, respectively, might have contributed towards the initiation of the tooth resorption process. Apical maturity of the root is an important factor which determines the result of the replanted tooth. Apical development at the time of replantation is significantly associated with tooth survival, since incisors with open apices showed lower survival compared with incisors with closed apices.^[10]^ Conversely, in the second patient (Case 2), only external root resorption was noted after a successfully accomplished root canal therapy. Taken together these findings indicate the role of the residual pulp tissue in the initiation and development of internal root resorption, whereas periodontal tissue injuries appear to in support external root resorption. Evidently, it is important to remove the entire necrotic pulp and complete the root canal therapy after tooth avulsion in order to prevent internal resorption.

The causes and underlying mechanisms for such resorptions remain unknown. There are numerous reports on the occurrence of internal^[6,11]^ and external^[8,12–15]^ tooth resorption as separate entities. However, for a tooth to be affected by both internal and external resorption at the same time is relatively rare. This report presents the exceptional case of a tooth resorbed from both within and outside, and discusses the pathological changes involved in the process.

Tooth resorption is mainly attributed to odontoclasts, which absorb dentin and cementum, and are located adjacent to the resorption areas. In the present report, several multinucleated odontoclasts were found in the resorption lacunae. The odontoclasts were smaller in volume than osteoclasts, and fewer in number. However, in some instances, multinucleated odontoclasts are not observed near the lacunae, probably because the resorption lacunae are in the quiescent period or due to the destruction of the odontoclasts during tissue preparation.

In a study by Sahara et al, it was reported that multinucleated dental pulp cells are similar to osteoclasts in morphology and function, and are capable of absorbing the 3 types of dental hard tissues. Osteoclasts and odontoclasts stem from hematopoietic cells in the marrow; however, osteoclasts can arise from vascular endothelial cells as well.^[16]^ In the present study, a large number of capillaries were noted in the granulation tissue surrounding the resorption zone in the Case 1 (Fig. 3F). The untimely removal of infected necrotic pulp tissue and damaged periodontal ligament vessels may have caused the undifferentiated mesenchymal cells in the granulation tissue to differentiate into odontoblasts and form reparative dentin. The cells may also differentiate into odontoclasts, although this remains to be confirmed.

There is comparatively more information regarding osteoclasts, whereas the exact mechanisms involved in odontoclast differentiation are still unknown. Ultrastructural studies have reported that odontoclasts and osteoclasts are similar in many ways; they have the same subcellular structures such as vacuoles, mitochondria and specific particle multinuclear. In addition, they are multinucleate, and contain brush-border cells and translucent zone. Similar to the osteoclasts, the odontoclasts induce apoptosis via the effect of diphosphonates, which can be inhibited by calcitonin.^[17]^ Thus, the combined application of calcitonin, diphosphonates and other drugs during the treatment of avulsed teeth may reduce the incidence of internal-external resorption. Osteoclast differentiation is mediated by a variety of molecules associated with bone resorption, such as RANK (Receptor Activator of Nuclear Factor kappa B) and its ligand (RANKL), which are expressed in odontoblasts, dental pulp cells and periodontal ligament cells.^[18–20]^ Osteoprotegerin (OPG) which can inhibit osteoclast differentiation, is expressed in periodontal ligament cells. Trauma, especially in avulsed teeth, results in the exposure of these factors from the injured periodontal ligament tissue. Thus, odontoblasts, dental pulp fibroblasts and periodontal ligament cells, through RANK, RANKL and OPG, mediate the differentiation of odontoclasts, which thereby influences the process of dental resorption. This might account for the mild external root resorption observed in Case 2 in the present study, whereby removal of necrotic pulp may have helped in reducing the production of the aforementioned factors.^[21]^

The expression of RANK, RANKL, and OPG are altered in odontoblasts, dental pulp cells, and periodontal ligament cells, thus influencing the precursors that differentiate into odontoclasts. They exert a direct effect on tooth resorption, suggesting that the constitutive expression of RANKL induces the spontaneous generation of osteoclasts (odontoclasts and cementoclasts) in the absence of osteotropic factors.^[22]^ The fact that permanent teeth are not resorbed under normal conditions, unlike bone, suggests that the mechanism involved in suppressing tooth resorption appear to be associated with OPG, which is strongly expressed in the dental pulp and periodontal ligaments.^[23]^ These results indicate that there should be a dynamic balance between both suppression and induction during tooth resorption. Otherwise, as seen in the 2 cases in this study, trauma and contamination of the periodontal ligament tissue may result in external resorption. However, a clear understanding of the factors that disturb the dynamic balance between suppression and induction of tooth resorption is lacking.

Osteoclasts and odontoclasts stem from hematopoietic cells in the marrow; nevertheless, osteoclasts can arise from vascular endothelial cells as well. An increasing number of CD14+ progenitor cells of osteoclasts (odontoclasts and cementoclasts) are produced in the blood from veins accumulating around dental pulp stem cells (DPSCs) and periodontal ligament stem cells (PDLSCs),^[23]^ resulting in the production of larger amounts of RANKL by DPSCs and PDLSCs. Moreover, under specific culture conditions such as hypoxia, vascular generation can be induced when co-cultured with DPSCs.^[24]^ A similar cellular environment and response might have prevailed in Case 1. A large number of capillaries were noted within the granulation tissue surrounding the resorption zone, and untimely removal of infected necrotic pulp tissue and damaged periodontal ligament vessels may have caused the undifferentiated mesenchymal cells to differentiate into odontoblasts and form reparative dentin (Fig. 3A, C).

Since tooth resorption has no symptoms, we do not know the time correlation between replantation and tooth resorption. The timing of observation of complications varied from 1 month to 2 years. Two types of resorption were detected, infection-related resorption in 20/32 teeth, while replacement resorption occurred in 7/32 cases.^[10]^

Current knowledge regarding the repair process of replanted teeth in humans after reimplantation has mostly been obtained from animal studies, observation of repair and healing after tooth extraction or apical surgery in humans, and cross-sections of extracted teeth. The findings of the present report contribute to this knowledge by presenting the histological findings of a tooth with extensive root resorption and apical periodontitis after having undergone a successful replantation treatment following avulsion a few years ago.

In summary, it is essential for the surgeon and the dentist to coordinate replantation and subsequent treatment strategies in patients with avulsed teeth. As demonstrated in this report, injury to the dental pulp tissue and periodontal ligament may be associated with the root resorption process, of the tooth, and it is therefore essential that the treatment of replanted teeth should involve effective management of these tissues.

## Author contributions

**Conceptualization:** Hongchen Sun, Xiangwei li.

**Data curation:** Huimin Liu, Xiaoxing Peng, Xiangwei li.

**Funding acquisition:** Xiangwei li.

**Methodology:** Huimin Liu.

**Supervision:** Xiaoxing Peng.

**Writing – original draft:** Huimin Liu.

**Writing – review & editing:** Huimin Liu, Xiaoxing Peng, Hongchen Sun, Xiangwei li.

Xiangwei li orcid: 0000-0001-7507-3616.
